# Non-neuronal cholinergic system delays cardiac remodelling in type 1 diabetes

This article has been retracted.

**DOI:** 10.1016/j.heliyon.2023.e17434

**Published:** 2023-06-19

**Authors:** Pujika Emani Munasinghe, Eng Leng Saw, Matthew Reily-Bell, Devin Tonkin, Yoshihiko Kakinuma, Martin Fronius, Rajesh Katare

**Affiliations:** a Department of Physiology, HeartOtago, University of Otago, 270, Great King Street, Dunedin, 9010, New Zealand; b Department of Bioregulatory Science, Graduate School of Medicine, Nippon Medical School, Tokyo, Japan

**Keywords:** Type 1 diabetes mellitus, Cardiovascular disease, Cardiac non-neuronal cholinergic system, Acetylcholine, Apoptosis, Cardiac function

## Abstract

**Aims:**

Type 1 diabetes mellitus (T1DM) is associated with increased risk of cardiovascular disease (CVD) and mortality. The underlying mechanisms for T1DM-induced heart disease still remains unclear. In this study, we aimed to investigate the effects of cardiac non-neuronal cholinergic system (cNNCS) activation on T1DM-induced cardiac remodelling.

**Methods:**

T1DM was induced in C57Bl6 mice using low-dose streptozotocin. Western blot analysis was used to measure the expression of cNNCS components at different time points (4, 8, 12, and 16 weeks after T1DM induction). To assess the potential benefits of cNNCS activation, T1DM was induced in mice with cardiomyocyte-specific overexpression of choline acetyltransferase (ChAT), the enzyme required for acetylcholine (Ac) synthesis. We evaluated the effects of ChAT overexpression on cNNCS components, vascular and cardiac remodelling, and cardiac function.

**Key findings:**

Western blot analysis revealed dysregulation of cNNCS components in hearts of T1DM mice. Intracardiac ACh levels were also reduced in T1DM. Activation of ChAT significantly increased intracardiac ACh levels and prevented diabetes-induced dysregulation of cNNCS components. This was associated with preserved microvessel density, reduced apoptosis and fibrosis, and improved cardiac function.

**Significance:**

Our study suggests that cNNCS dysregulation may contribute to T1DM-induced cardiac remodelling, and that increasing ACh levels may be a potential therapeutic strategy to prevent or delay T1DM-induced heart disease.

## 1 Introduction

Type 1 diabetes mellitus (T1DM) affects approximately 10% of the 537 million adults living with diabetes worldwide in 2021 [1]. Cardiovascular disease (CVD) is the leading cause of mortality in individuals with T1DM [2,3]. Huxley et al. [4] conducted a meta-analysis and reported that men with T1DM have a mortality ratio of 5.7 attributed to CVD, while women have a mortality ratio of 11.3. The mechanisms underlying CVD in T1DM are multifactorial, involving reduced oxygen availability [5], excessive free fatty acid accumulation [6], impaired glucose metabolism [7], autonomic neuropathy [8], and impaired cardiac function [9].

Of these mechanisms, autonomic neuropathy resulting from nerve damage has received little attention. Dysregulation of the sympathetic or parasympathetic nervous system is associated with fatal consequences [10]. The heart contains both a neuronal cholinergic system and a non-neuronal cholinergic system (NNCS) [11], both of which produce and release the neurotransmitter acetylcholine (ACh) [11]. The neuronal system releases ACh via muscarinic receptors, while the NNCS releases ACh as an auto-/paracrine mediator. The activity of the cardiac NNCS (cNNCS) is associated with the activation of the pro-survival Akt signalling cascade, which is important for normal heart function [[12], [13], [14]].

Recently, we provided evidence for a role of the cNNCS in the hearts of individuals with type 2 diabetes. Dysregulation of the cNNCS proteins was observed in both human type 2 diabetic individuals and in an animal model of type 2 diabetes [15]. Nonetheless, the involvement of the cNNCS in T1DM and its associated CVD remains uncertain. To address this question, we used an animal model of T1DM induced by administering streptozotocin (STZ) to investigate the role of the cNNCS in T1DM. Interestingly, transgenic mice with cardiac-specific overexpression of choline acetyltransferase (ChAT), a crucial enzyme in acetylcholine (ACh) synthesis, exhibited prevention of cNNCS dysregulation in the T1DM heart. Importantly, this was associated with preservation of microvessels and cardiac function, indicating that the cNNCS indeed plays a role in T1DM. Consequently, promoting elevated levels of cardiac ACh through an activated cNNCS might present a promising approach for averting T1DM-induced cardiac dysfunction.

## 2 Materials and methods

### 2.1 Ethics

The Animal Ethics Committee from the University of Otago (AEC number 25/12) and Nippon Medical School, Japan, approved the use of animals for this study.

### 2.2 Induction of T1DM in ChAT transgenic mice

A transgenic mouse model that is characterised by the overexpression of the murine *Chat* gene (ChAT-Tg) in the heart was utilized for this study. ChAT-Tg mice are developed in our laboratory in collaboration with Professor Masayuki Tsuda, Institute for Laboratory Animal Research, Kochi University, Japan, and have been well characterized in previous studies [[15], [16], [17], [18], [19]]. To induce T1DM, 12-week-old ChAT-Tg mice and their wild-type litter controls were given an intraperitoneal injection of STZ at 50 mg/kg/day for 5 days [20,21]. Our previous studies have extensively characterized the development of cardiac dysfunction in this model of T1DM [21,22]. The development of diabetes was confirmed using Comber Test® E strips to measure the glucose level in the urine before recruiting the mice to the experimental group (206 ± 24 mg/dL in T1DM mice and 200 ± 12 mg/dL in ChAT-Tg). Mice with urine glucose levels of 50 mg/dL and above were considered diabetic or hyperglycemic and included in the study. Wild-type mice injected with a buffer (without STZ) vehicle served as non-diabetic controls. Low dose streptozotocin has evolved into a preferred method for inducing T1DM in animal models, as it leads to a gradual onset of diabetes. This method has the advantage of mimicking the slow onset of human type 1 diabetes, unlike high dose streptozotocin which rapidly destroys beta cells and causes severe inflammation and toxicity. This has made low dose STZ a more reliable and efficient model for studying the pathophysiology of type 1 diabetes [23,24].

### 2.3 Measurement of cardiac function

Left ventricular function was measured in animals at 4, 8, 12, and 16 weeks post STZ injection using a pressure-volume (PV) catheter [25]. Briefly, while the animals were under isoflurane anesthesia, a small incision was made in the abdominal cavity to insert the PV catheter through the diaphragm into the apex of the heart. Isoflurane was chosen as the anesthesia due to its negligible impact on heart rate, as observed in our prior investigations. Notably, the brief exposure to isoflurane during this procedure did not result in any discernible effects on the heart. The PV catheter was then connected to an ADVantage PV system control box (Transonic Systems) and a data acquisition system (iWorx system). Hemodynamic parameters were recorded using LabScribe2 software (iWorx system). After the functional analysis, the animals were humanely euthanized, and heart samples were collected and preserved for subsequent molecular and histological analyses.

### 2.4 Total protein extraction and Western blot analysis

Total protein was extracted from the frozen tissue sample after homogenizing the tissues with RIPA buffer supplemented with a 1% protease cocktail inhibitor. Ten micrograms of total protein were separated by SDS-PAGE and transferred to the PVDF membrane. The membrane was probed with primary and secondary antibodies against key proteins associated with cNNCS and cell survival cascade. Details of the primary and secondary antibodies used are provided in the online supplement (Supplementary Table 1). The chemiluminescence signal to visualize the proteins was captured by a Syngene Pxi imaging system (USA). Band density was analyzed using ImageJ software (NIH). The target protein was normalized to the band intensity of a prominent band between 75 kDa and 100 kDa from Ponceau S stained blot (total protein expression level) [26] and expressed as a ratio of the target to total protein ratio [27].

### 2.5 Cardiac ACh measurement

Cardiac ACh levels were determined by HPLC [15] and using a commercially available Choline/Acetylcholine assay kit (ab65345, Abcam) [28]. For HPLC, the left ventricle was harvested and homogenized in 0.1 M perchloric acid containing 0.1 mM AChE inhibitor physostigmine and an internal control of isopropylhomocholine (5 × 10-7 M). The tissue lysate was centrifuged, followed by filtration using a 10 K centrifugal filter column (Amicon Ultra, UFC501096). Then, 10 μL of the filtered lysate was injected into an HPLC system (HTEC-500; Eicom, Japan). For the measurement of ACh using assay kit, 10 mg of tissue was homogenized with Choline Assay Buffer. Following centrifugation, the supernatant was collected and used to measure the level of total choline and free choline. The concentration of ACh was then determined as the difference between total and free choline.

### 2.6 Immunohistochemical analysis for cardiomyocyte apoptosis and fibrosis

As a measure for cardiac damage apoptotic cardiomyocytes were detected and quantified in 7 μm thick myocardial cryosections using terminal deoxynucleotidyl transferase dUTP nick end labelling (TUNEL) staining using the commercially available kit (Click-iT™ Plus TUNEL Assay Kits for In Situ Apoptosis Detection, C10617, ThermoFisher Scientific, New Zealand) following our previously published protocol [29]. Following TUNEL staining, sections were probed with biotin-conjugated cardiac Troponin I Type 3 mouse monoclonal antibody (1:100 dilution, NB110–2546B, Novus Biologicals, USA) to label cardiomyocytes and counterstained with Alexa Fluor 488 streptavidin (1:1000 dilution, S32354, ThermoFisher Scientific, New Zealand). Images were captured at 200× magnification using an Olympus B×51 fluorescence microscope. Data are expressed as the percentage of TUNEL positive cardiomyocytes nuclei.

To determine the level of fibrosis, sections were stained with 0.1% direct red 80 (Sigma Aldrich)/Picric acid solution (Sigma Aldrich). A whole ventricular section image was captured using an Olympus AX70 microscope fitted with a polarized lens. Data are expressed as a percentage of the fibrotic area by normalizing the polarised tissue area to the total cardiac tissue area and fold changes in the fibrotic area compared to the non-diabetic group of the corresponding time point. All data were analyzed using Image J software (NIH, USA).

### 2.7 Statistical analysis

Sample size was determined based on our earlier studies using type-1 diabetic mouse model [21,22,30]. GraphPad Prism 8.0.2 software (GraphPad Prism® Version 8.0.2, GraphPad Software, Inc.) was used for all statistical analyses. Shapiro-Wilk test was used to test the normality of data distribution. When the normality test failed, the non-parametric Kruskal-Wallis test was used to compare the expression levels between the study groups at a specific time point. Statistical test used for individual analysis is described in the figure legends. Comparisons were made between the study groups at a given time only for Western blot experiments, as it was impossible to run all the samples in the same blot. A *P*-value <0.05 was considered to be statistically significant for all comparisons.

## 3 Results

*All the uncropped original blot images are presented as*Supplemental Figures.

### 3.1 T1DM induced dysregulation of cNNCCs components in the heart, which was partially restored by overexpression of ChAT

Western blot analysis showed significant downregulation of ChAT (Fig. 1A& Supplemental Fig. 1) at 4-weeks and 16-weeks after T1DM induction in comparison to non-diabetic animals. There was also a significant downregulation of CHT-1 at 16-weeks after T1DM induction (Fig. 1B& Supplemental Fig. 2). In animals with T1DM no changes in the expression of AChE (Fig. 1C& Supplemental Fig. 3) and VAChT (Fig. 1D& Supplemental Fig. 4) were observed. Importantly, the observed changes in the expression of NNCS proteins were associated with a marked reduction in cardiac ACh levels (Fig. 1E & F).

**Fig. 1:** Representative Western blot images and quantitative scatter plot bar graphs showing the expression of Choline Acetyltransferase (ChAT, **A**), choline transporter-1 (CHT-1, **B**), Acetylcholine esterase (AChE, **C**), vesicular ACh transporter (VAChT, **D**) and type-2 muscarinic ACh receptor (M_2_AChR, **G**) at different time points after induction of type 1 diabetes mellitus (T1DM). Shapiro-Wilk test was used to test the normality of data distribution. Two-way analysis of variance yielded a significant interaction effect for ChAT (*F*(6, 60) = 5.76, p < 0.0001) and CHT-1 (*F*(6, 61) = 3.96, p = 0.0021) and a non-significant interaction for VAChT (*F*(6, 62) = 1.09, p = 0.374), AChE (*F*(6, 59) = 1.78, p = 0.119) and M_2_AChR (*F*(6, 60) = 0.96, p = 0.463). The non-parametric Kruskal-Wallis test was used to compare the expression levels between the groups. Data are presented as the ratio of the target protein to total protein as visualized by ponceau staining and are median with interquartile range. n = 6 in each group. All the western blots are repeated at least two independent times. For ChAT expression, although all the samples were run in the same blot (as shown in Supplemental Fig. 1), due to the strong expression of ChAT in the transgenic heart, the blots were first exposed to image ChAT expression in the transgenic heart, followed by exposing only the ND and T1DM groups for a longer time. A dotted line indicates this between the ND and T1DM group and the ChAT-Tg-T1DM group. **E & F.** Scatter plot bar graphs showing ACh levels in the study groups measured using HPLC (**E**, data presented as μmol/gram of heart tissue) and ACh assay kit (**F**). Shapiro-Wilk test was used to test the normality of data distribution. A two-tailed unpaired *t*-test was used to calculate the difference in ACh measured by HPLC (**E**) and the non-parametric Kruskal-Wallis test was used to compare the difference between the groups in ACh measured using the assay kit (**F**). Two-way analysis of variance yielded a significant interaction effect for ACh by assay kit (*F*(2, 17) = 4.04, p = 0.037). Data are presented as nmol/gram of total protein ratio of the target protein to total protein as visualized by ponceau staining and are median with interquartile range). n = at least 5 in each group. *P < 0.05, **P < 0.01 and ****P < 0.0001.

In ChAT-Tg animals, as expected, there was a marked increase in the expression of ChAT in at all the time points detected (Fig. 1A& Supplemental Fig. 2), which was associated with a significant increase in ACh levels (Fig. 1F). In these animals, and in contrast to the wild type animals, CHT-1 expression was unchanged (Fig. 1B& Supplemental Fig. 1), while in agreement with wild type no effect on VAChT was observed (Fig. 1D & Supplemental Fig. 3). Interestingly, ChAT overexpression induced significant downregulation of AChE at 16-weeks post DM induction (Fig. 1C& Supplemental Fig. 3).

While T1DM did not affect M_2_AChR expression, ChAT overexpression significantly increased the expression of M_2_AChR at 8, 12 and 16 weeks post T1DM induction compared with wild type, and specifically at 16 weeks compared with T1DM (Fig. 1G& Supplemental Fig. 5).

### 3.2 ChAT overexpression restored T1DM induced downregulation of the pro-survival cascade

A potential mechanism of how cNNCS mediates its effects is through the pro-survival Akt pathway [15,31]. In Western blot analysis we were able to detect a significant downregulation of phosphorylated Akt from early stages of T1DM (Fig. 2A& Supplemental Fig. 6). This was associated with significant downregulation of Bcl-2 a downstream target of Akt (Fig. 2B& Supplemental Fig. 7). Bcl-2 is an anti-apoptotic protein that plays a vital role in the cross-talk and coupling of the Akt pathway to reduce apoptosis, thereby reducing oxygen demand in the heart [32]. Thus, the changed expression of cNNCS proteins seems to correlate with reduced function of the pro-survival Akt pathway and elevated apoptosis.

**Fig. 2:** **A&B.** Representative Western blot images and quantitative scatter plot bar graphs showing the expression of pAkt and Akt (**A**) and Bcl-2 (**B**) at different time points after induction of type 1 diabetes mellitus (T1DM). Shapiro-Wilk test was used to test the normality of data distribution. Two-way analysis of variance yielded a significant interaction effect for Bcl-2 (*F*(6, 60) = 2.54, p = 0.0295) and a non-significant interaction for pAkt/Akt (*F*(6, 59) = 0.866, p = 0.525). The non-parametric Kruskal-Wallis test was used to compare the expression levels between groups. Data are presented as the ratio of the target protein to total protein as visualized by ponceau staining and are median with interquartile range. n = 6 in each group. All the western blots are repeated at least two independent times. **C.** Representative fluorescent microscopic images and quantitative scatter plot bar graphs showing TUNEL positive cardiomyocytes. Arrowheads points the apoptotic cell. Shapiro-Wilk test was used to test the normality of data distribution. Two-way analysis of variance yielded a significant interaction effect (*F*(2, 30) = 3.83, p = 0.0331) The non-parametric Kruskal-Wallis test was used to compare the TUNEL positive cardiomyocytes between the groups. Data are represented as TUNEL^+^ cardiomyocytes/field and are mean ± SEM. n = 6 in each group. Scale bars are 50 μm.

However, both Akt and Bcl-2 expression were normal in the ChAT-Tg heart (Fig. 2A&B& Supplemental Fig. 6&7), suggesting reduced apoptotic cell death. Reduced apoptosis was further observed with the TUNEL assay, showing a significant reduction in TUNEL positive cardiomyocytes in the ChAT-Tg heart at 16 weeks after T1DM induction (Fig. 2C& Supplemental Fig. 8).

### 3.3 ChAT overexpression reduced abnormal ventricular and vascular remodelling in the T1DM heart

Sirius red staining showed a marked increase in cardiac fibrosis in the T1DM heart at both early and late time points (8.3 ± 0.96 and 22.8 ± 3.54-fold increase at 4- and 16-weeks respectively after STZ injection compared to ND, Fig. 3A-C& Supplemental Fig. 9), which was significantly prevented in the diabetic ChAT-TG heart (0.97 ± 0.003 and 1.62 ± 0.007-fold decrease at 4-, and 16-weeks respectively after STZ injection, Fig. 3A&B). Furthermore, we analyzed the density of capillaries and arterioles. In T1DM a marked decrease in the capillary density at 16 weeks was observed (Fig. 3C&D& Supplemental Fig. 10), which was prevented in the ChAT-Tg heart (Fig. 3C&D). Interestingly, the capillary density in ChAT-Tg hearts was increased at 12-weeks after T1DM induction compared to ND and T1DM hearts (Fig. 3C&D). Regarding the arteriole density, no significant difference was detected (Fig. 3C&E), although the ChAT-Tg heart showed a small increase in arteriole density at 12 and 16 weeks but this was not significant (Fig. 3E).

**Fig. 3:** **A-C.** Representative microscopy images captured with polarised lens (**A**) and the quantitative scatterplot bar graphs showing the fold-changes in the fibrotic area compared to ND of the corresponding time point (**B**). Scale bars are 500 μm. Shapiro-Wilk test was used to test the normality of data distribution. Two-way analysis of variance yielded a significant interaction effect (*F*(2, 30) = 13.82, p < 0.0001) The non-parametric Kruskal-Wallis test was used to compare the TUNEL positive cardiomyocytes between the groups. n = 6 in each group. **C-E.** Representative confocal microscopy images (**C**) and the quantitative scatterplot bar graphs show the capillaries (isolectin, green, **D**) and arterioles (α-smooth muscle actin (α-SMA), red, arrowhead **E**) at different time points. Shapiro-Wilk test was used to test the normality of data distribution. Two-way analysis of variance yielded a significant interaction effect for capillaries (*F*(6, 55) = 5.232, p = 0.0003) and arterioles (*F*(6, 56) = 3.006, p = 0.0129). Tukey's multiple comparisons test was used to compare the capillaries and arteriole density between the groups. n = 6 in each group. Data are represented as the number of capillaries (**D**) and arterioles (**E**) per mm^2^ and are mean ± SD. (For interpretation of the references to colour in this figure legend, the reader is referred to the Web version of this article.)

### 3.4 ChAT overexpression prevented impairment of cardiac function in the T1DM heart

Functional analysis revealed diastolic and systolic dysfunction as early as four weeks after T1DM induction, as evidenced by increased left ventricular (LV) end-diastolic volume (Fig. 4A), increased LV end-systolic volume (Fig. 4B) and reduced ejection fraction (Fig. 4C). Moreover, T1DM reduced LV end-systolic pressure at 16-weeks after T1DM induction (Fig. 4D), while there was no difference in end-diastolic pressure (Fig. 4E). With the exception of LV end-diastolic pressure, these impairments were not observed in ChAT-Tg hearts indicating that elevated ACh has cardioprotective effects. This is likely due to the preservation of pro-survival cascades, which prevented abnormal ventricular and vascular remodelling (Fig. 4A–E). There was a trend towards reduced heart rate in the diabetic group; however, overexpression of ChAT had no further effect (Fig. 4F).

**Fig. 4:** Quantitative bar graphs showing the cardiac function measured using a pressure-volume catheter at different time points. EDV – Left ventricular (LV) end-diastolic volume; ESV – LV end-systolic volume; EF – LV ejection fraction; ESP – LV end-systolic pressure; EDP – LV end-diastolic pressure; HR – heart rate. Shapiro-Wilk test was used to test the normality of data distribution. The non-parametric Kruskal-Wallis test was used to compare the differences between the groups. N = 8–9 in each group.

## 4 Discussion

Our study identified dysregulation of the cNNCS and reduced ACh levels in T1DM that were associated with impaired cardiac function. Our findings regarding the role of the cNNCS in T1DM are consistent with a previous study that showed a significant reduction in ChAT expression in T2DM hearts[ [15]. While we observed downregulation of ChAT as early as 4 weeks after T1DM induction, there was no significant difference in expression patterns at 8 and 12 weeks compared to ND counterparts. The time-dependent change in expression levels is likely due to the compensatory response of the heart to acute glycaemic stress, as reported in our previous study, which showed upregulation of pro-survival factors in response to glycaemic stress as part of a compensatory mechanism [22].

We also observed a significant downregulation of CHT-1 in the late stage of diabetes, indicated decreased ACh synthesis in the diabetic heart [33]. This is supported by a previous study showing reduced ACh synthesis in mouse cardiomyocytes treated with the CHT-1 inhibitor hemicholinium-3 [34]. Newman et al. reported a significant alteration in heart rate variability in individuals with the CHT1 “3′UTR gene” polymorphism, indicating a role for CHT-1 in regulating cardiac function [35]. ChAT, CHT-1 and VAChT are required for the production and secretion of ACh. In our study ChAT overexpression prevented the downregulation of CHT-1 but did not affect the expression of VAChT. This is in agreement with a study from Matsuo et al. who reported activation of CHT-1 but not VAChT in a neuroblastoma cell line that overexpressed ChAT [36]. Our findings suggest that ChAT overexpression induced translational activation of CHT-1 in the diabetic heart.

Our study uncovered another interesting finding that could explain the increased ACh levels in ChAT-Tg hearts. This could be possibly due to the downregulation of AChE. AChE's primary function is to hydrolyze ACh to acetic acid and choline [37]. However, reduced AChE leads to a decrease in the breakdown of ACh, thereby increasing both the level and duration of ACh action [38]. Although the reason for reduced AChE expression in ChAT Tg hearts is unclear, it may be due to a mismatch between increased ACh level and the available AChE enzyme. Further investigations to identify the exact reason will be of interest.

Both T1DM and T2DM are linked to the progressive loss of cardiomyocytes [22,29,39] and increased fibrosis [40]. Kuethe et al. showed an 85-fold increase in cardiomyocyte apoptosis in the heart tissue collected from patients with T1DM and cardiomyopathy [41], which was also evident in our study, showing a significant increase in cardiomyocytes apoptosis from an early stage of diabetes. Increased apoptotic cell death in the diabetic heart is directly related to the downregulation of the pro-survival Akt pathway in the T1DM heart [22]. This is likely due to a lack of insulin in T1DM, as insulin is a direct activator of the Akt pathway and its downstream targets such as Bcl-2 [42,43]. Moreover, increased reactive oxygen species and production of advanced glycation end products as a consequence of hyperglycaemia also directly impair the Akt pathway [44,45]. Previous studies have shown that ACh induced activation of PI3K/Akt/HIF1α/GLUT-4 signalling cascade through its interaction with M_2_AChR in the cardiomyocytes [15,16,46,47]. Further activation of the Akt signalling pathways increases the availability of hypoxia-inducible factor 1-alpha (HIF-1α) which in turn activates pro-angiogenic endothelial nitric oxide synthase (eNOS) [16,46,47]. In our study, ChAT overexpression prevented vascular rarefaction in the diabetic heart, which is likely through the Akt or nitric oxide (NO)-mediated activation of HIF-1α, although the direct association between ChAT overexpression and activation of HIF-1α requires confirmation.

There are a few limitations to this study. First, we used only male mice for this study to avoid the effects of estrogen, as our previous study showed activation of NNCS by estrogen [48]. However, diabetes disproportionately affects females [21]. Therefore, future studies should include female animals. Secondly, the ChAT-Tg mice have increased ACh levels since birth, while T1DM in humans occurs at a later age. Therefore, alternative methods to increase ACh levels after the development of diabetes are important to translate this therapeutic approach to the clinic. One possibility is to use the pharmacological approach to inhibit the breakdown of ACh. Cholinesterase inhibitors are clinically used for the treatment of Alzheimer and dementia symptoms [49]. A recent propensity score matching study demonstrated lower incidence of new-onset heart failure in patients with Alzheimer's disease prescribed with cholinesterase inhibitors after 10-years follow up [50]. Therefore, it will be interesting to test whether cholinesterase inhibitors may have beneficial effects in delaying the onset of diabetic heart disease. Thirdly, it will also be important to determine if T1DM affects other cNNCS components, such as electrogenic cation transporters (OCTs) and butyrylcholinesterase (BChE), which are complementary to AChE [51]. This is important because some of the tested cNNCS components were affected in diabetes in this study.

In conclusion, this study sheds light on the role of the cholinergic anti-inflammatory pathway in the context of type 1 diabetes-induced cardiac dysfunction. The findings suggest that dysregulation of the cNNCS and reduced ACh levels are associated with impaired cardiac function, and increasing ACh levels in the heart can prevent these effects. The study also provides insights into the time-dependent change in expression level of ChAT and CHT-1 and the compensatory response of the diabetic heart. Additionally, the study highlights the potential of ChAT overexpression as a therapeutic approach to prevent cardiomyocyte apoptosis, interstitial fibrosis, and vascular rarefaction in type 1 diabetic hearts. Despite a few limitations, the study provides a proof-of-concept for the use of ChAT overexpression to increase ACh levels, which could be beneficial to the T1DM heart. Future studies can further explore the role of other cNNCS components, determine alternative methods to increase ACh levels after diabetes development, and evaluate this therapeutic approach's translation to the clinic.

## Author contribution statement

Pujika Emani Munasinghe, Eng Leng Saw, Matthew Reily-Bell, Devin Tonkin: Performed the experiments; Analyzed and interpreted the data; Contributed reagents, materials, analysis tools or data; Wrote the paper.

Yoshihiko Kakinuma, Martin Fronius, Rajesh Katare: Conceived and designed the experiments; Analyzed and interpreted the data; Contributed reagents, materials, analysis tools or data; Wrote the paper.

## Funding statement

Assoc Prof Rajesh Katare was supported by 10.13039/501100001509Royal Society Te Apārangi (18-U00-01-CSG).

Yoshihiko Kakinuma was supported by 10.13039/501100001691Japan Society for the Promotion of Science (16K0856), 10.13039/501100004330Smoking Research Foundation (2019-22).

## Data availability statement

Data included in article/supp. material/referenced in article as well as detailed protocols are available upon request to the corresponding authors.

## Declaration of competing interest

The authors declare the following financial interests/personal relationships which may be considered as potential competing interests:Rajesh Katare reports financial support was provided by 10.13039/501100001509Royal Society of New Zealand. Yoshihiko Kakinuma reports financial support was provided by 10.13039/501100001691Japan Society for the Promotion of Science. Yoshihiko Kakinuma reports financial support was provided by 10.13039/501100004330Smoking Research Foundation.
